# A Study of Cloud-Based Remote Clinical Care Technology

This article has been retracted.

**DOI:** 10.1155/2021/8024091

**Published:** 2021-12-06

**Authors:** Bo Lin, Wei Huang

**Affiliations:** ^1^Department of Fundamental Nursing, West Anhui Health Vocational College, Lu'an, Anhui Province 237005, China; ^2^Intensive Care Unit, Affiliated Hospital of West Anhui Health Vocational College, Lu'an, Anhui Province 237005, China

## Abstract

This paper uses cloud computing to build and design remote clinical care technology, and the study refines the evaluation approach for the elements and builds an evaluation prototype for the strategy, uses service design theory to improve the design of the service part of the assistive system, summarizes the list of requirements based on system design and service design, and designs a service design prototype. Through design practice, the detailed design of the software interaction interface and the auxiliary product of the care assistance system based on the prototype are investigated. Based on the user perspective, the strategy of meeting user expectations and improving user information literacy is proposed; based on the social network perspective, the strategy of establishing a long-term mechanism for smart medical operation and improving the information interaction network environment is proposed; and based on the system service perspective, the strategy of optimizing the system function design and innovating the service model is proposed. Compared with the traditional written patient handover, the application of MNIS under cloud computing can significantly shorten the handover time of surgical patients, improve the standardized rate of surgical safety verification execution and the qualified rate of nursing documents, while the rate of standardized application of prophylactic antibiotics is also significantly higher than that of the control group. The questionnaire survey of nursing staff in the operating room showed that clinical nursing staff was generally satisfied with the clinical application of MNIS under cloud computing, with an average satisfaction score of 64.5 to 11.3, and an average score of 3.58 to 0.54 for each item. Among them, pre-application training of MNIS, departmental support for MNIS, and its ease of verification in surgical patients were the three main factors favoring the clinical application of MNIS in the operating room with cloud computing, while barriers to wireless network connectivity, inconvenient PDA input, and small screen size were the three main drawbacks affecting its application. The determined clinical evaluation index system of MNIS in the operating room is innovative, which not only includes clinical care indicators but also covers general hardware and software indicators, which can effectively reflect the practical application capability of mobile terminal clinical and user experience feelings, and the evaluation index system is comprehensive.

## 1. Introduction

Nursing information competency is a combination of knowledge, skills, and attitudes that match the prescribed level of nursing practice and are demonstrated in various nursing information activities, and nursing information competency mainly covers nursing information competency and nursing information practice competency [1]. Nursing staff must have sufficient information competence to actively participate in and lead the development of hospital information technology. With the continuous development of remote nursing, mobile nursing, and intelligent nursing, the role of NIS no longer was limited to transcription, transmission, and transcription of medical orders, and the function of NIS has changed from traditional disease-care-centered to nursing support and health care, which requires nurses' computer application ability, computer software management ability, nursing information awareness, and management ability increasingly [2]. Therefore, innovative practice behaviors in nursing information systems require nurses to have the above information competencies. Innovative competencies of nurses are the ability of clinical nurses to proactively seek and develop new methods, techniques, and appliances for health promotion, pre-squared diseases, and improved quality of patient care, and to apply innovations to their work through teamwork and reasonable channels of support. The innovative behavior of nurses is the external manifestation of innovative ability, and the innovative behavior of nurses includes idea generation, idea support, and idea realization, and in different stages of innovative behavior, the innovative behavior of nurses is related to individual traits and collective atmosphere, where the innovative use behavior of NIS is related to individual traits of innovative consciousness, willingness to innovate, IT knowledge, and skills [3]. Eliminate the uncertainty of the information recipient's understanding of things. Traditional information transmission methods mainly include sensory transmission, written transmission, and telecommunications transmission. The speed of sensory transmission is faster, but the information is more difficult to store. In summary, nurses' innovative use behavior of NIS should be based on information competence and innovation ability, and nurses should have the courage and methods to reform the existing functions of the system, identify problems from nursing practice, and use IT to solve clinical problems to truly promote the change of their innovative use behavior, i.e., nurses' innovative use behavior of NIS needs both nursing information competence and innovation ability [4].

The behavior of nurses in the process of using information systems is measured by problem and strategy formulation, participation in innovative behaviors, and continuously improving information system module functions and developing new system functions or ways of using the system by giving feedback on problems and collaborating with relevant departments to propose improvement strategies [5]. However, the implementation of the current HIS is based on the operation of computer terminals in fixed places, so medical and nursing staff sometimes cannot give timely diagnosis and treatment advice when making rounds or operating at the patient's bedside; nursing staff needs to fill in relevant data and information in writing during the “three checks and seven pairs” at the bedside; in addition, some patient health information also needs to be collected clinically by medical and nursing staff and then input into the computer terminal [6]. In addition, some patient health information needs to be clinically collected by medical staff and then input into the computer terminal. Even in domestic tertiary hospitals where information technology construction is relatively advanced, medical and nursing staff still need to complete a considerable number of written medical documents manually, which not only wastes medical costs and human resources but also easily leads to errors when repeatedly transcribing data entered into patient information, resulting in errors in relevant medical information, which not only affects the consistency of data and information but also easily induces unnecessary medical disputes in the current medical environment.

MNIS under cloud computing platform can be free from the current hardware constraints on medical care information processing system and can call relevant data resources at any time in medical care, including the patient's complete medical history resources dating several years ago, or when encountering rare problems in medical care that are difficult to explain or solve, the relevant database information can be called for comparison and identification. The MNIS under the cloud computing platform enables nursing staff to process patient-related information in a more timely and efficient manner, while spending more time on patient care, truly realizing the “patient-centered” requirement. The medical staff can enter health information, check medical prescriptions and medication records, charge billing, as well as the patient's current complaints and signs into the mobile terminal at the patient's bedside and save them in the information system, thus avoiding repeated transcriptions and assisting the medical staff to execute the relevant important points of diagnosis and care operations on time, thus reducing the occurrence of medical errors. The operating room, as a relatively centralized department for medical care operations, is a multidisciplinary and multi-departmental centralized platform with more stringent care requirements. As an important platform department of the hospital, the operating room is a decisive core department to ensure the safety of patient surgery and provide quality perioperative care to patients, and it can be said that the safety and quality of nursing care in the operating room is one of the fundamental conditions for the quality of hospital operation. Community influence refers to the extent to which the interpersonal relationships and social structure around users affect their use of information systems or technologies; convenience conditions refer to the extent to which factors such as economic level, institutional policies, innovative technologies, and application environments support users' use of information systems or technologies. In the current era of big data, digital management has become the development direction of modern operating room construction, as well as an important part of digital hospital construction. According to the national diagnosis and treatment technical specifications and surgical safety target requirements, safe care involves not only the management of the surgical process, but it also involves all aspects of the perioperative period, so the comprehensive control and fine management of all these contents need a lot of information and data support.

## 2. Current Status of Research

Since the concept of cloud computing has only been proposed for about 10 years, and the health cloud is still being explored, the impact of the existing private clouds on healthcare management has not yet been highlighted, and its impact on nursing management is still not reported in detail. The current research on nursing information technology is more focused on MNIS application research, which is only an important part of the cloud computing platform [7]. The operating room is a multidisciplinary and multi-specialist platform for performing surgery or resuscitation of patients with acute and critical illnesses, and its safe and effective operation is crucial to the overall operational efficiency of the hospital. In the current healthcare environment, one of the important cores of surgical nursing is nursing safety [8]. Nursing safety requires that nursing staff at all levels to follow strict systems and standard practices, ensure that medical orders are carried out accurately, and develop and implement individualized and appropriate care plans so that patients can fully benefit from their treatment and recovery. Information technology in surgical care theoretically helps to improve the quality and efficiency of care and enhances nursing safety [9]. At present, due to security and privacy concerns, public health clouds are not fully developed but more often limited to private clouds within individual organizations, i.e., hospital cloud computing platforms, which serve as support platforms for internal hospital operations and are not open to the public [10]. For example, Taiwan Taichung Renmin Hospital's network application cloud image data center (CIDC) platform; patients can visit any hospital in the cloud, image data can be uploaded by Taichung Renmin General Hospital physicians to give consultation and diagnosis, thereby shortening patient consultation time, and improving the quality of medical care [11]. It has effectively improved the speed, efficiency, and quality of medical services.

Some scholars, on the other hand, suggest the establishment of specialized hybrid clouds, such as the establishment of an advanced 3D analysis master-slave system integrated with cloud computing for cardiovascular image database, which helps clinicians to evaluate the surgical outcome during endoluminal aortic valve replacement [12]. The establishment of a cloud computing platform also helps medical diagnosis, such as for lung nodules, by storing huge amounts of relevant medical data in the cloud platform, so that clinicians can quickly and accurately make a diagnosis by comparing and referring to existing databases through cloud computing. It is considered that the core content of smart medical includes the intelligent perception of medical objects, standardized disposition of medical processes, and integration of medical objects and medical processes through interconnection technology, and based on intelligent management of people, objects, and equipment, the medical IoT application model is studied from the medical service application model, medicine management application model, and medical device management application model, and the internal hospital medical [13]. The process of the digital collection, processing, storage, transmission, and sharing of medical information, equipment information, drug information, personnel information, and management information within the hospital is designed. After sorting out the status of research on smart medical systems, it was found that there is a lack of empirical research on the impact of smart medical system applications on patient satisfaction with medical care in China; so the mechanism of the impact of smart medical system applications on patient satisfaction with medical care was explored, and it was concluded that self-efficacy and perceived usefulness can positively affect patient satisfaction with medical care [14].

This MNIS architecture uses a combination of a data flow style and a warehouse style. Each node in the data flow style has its input and output pathway, and the data flow input is processed internally and then the corresponding data flow results are output. This process enriches the data by adding information step-by-step, which makes the software well hidden, highly cohesive, and low coupled, and facilitates the statistical analysis of the system. And, the warehouse style is a data-centric system that is practical for data storage, analysis, maintenance, and application.

## 3. Analysis of Remote Clinical Care Technologies for Cloud Computing

### 3.1. Analysis of Remote Clinical Care Cloud Computing Methods

It is a streamlined scheduling model, which is prototyped for distributed programming and efficient data scheduling tasks, in information systems, to facilitate the characteristics of computer parallelism, and it is necessary to constitute a common model as if the use of multi-threaded, multi-process processing, cloud computing technology is an important basis for the development of cloud computing, so as to focus on efficient programming models, in the case of large-scale data programming [15]. The parallelism of processes is major when it comes to large-scale data programming, as it can demonstrate efficient scheduling capabilities and can handle huge-scale data sets. Accurately meeting the diverse and multi-level health needs of patients is a nursing service model with development potential. In-hospital care focuses on optimizing the nursing process online. For example, the use of PDA enables nursing staff to identify patients, record the nursing process, collect physical data, query drug usage, and enter consumables charges. When the command is executed, the data area is divided and then the result of data processing is summarized to finalize the program, so that the programmer focuses more on the process of writing the program and does not pay attention to how the background is running; if the platform of cloud computing can be played, this will be the intuitive feedback of the performance of the whole cloud platform. The distributed system can store a large amount of data, guarantee data security, provide reliable storage, test IO throughput capacity, and expand its indicators. The number of users of the cloud computing system is mostly to improve its ability to handle data and the ability of computing; it must have safe data processing capacity and storage capacity. Traditional computer technology takes the form of direct-connected storage, network access storage. Traditional information processing is difficult to manage in terms of maintenance and management, with dedicated hardware in the branch office in-network access servers. Cloud computing data storage room can be extended into a distributed file system, using a simple storage device model. After meeting the daily security requirements, in many of the client distribution systems, you can achieve storage performance.

(1) $$\begin{array}{c} Q_{N}\left(w\right)={\sum_{i,j}\left(1+P_{ij}\right)}^{3}+\left(m_{i}-m_{j}\right). \end{array}$$

When mass data calculation is carried out on a large scale, data in the process of analysis, cloud computing data for processing, must have a powerful function of processing data. In data management, massive data are very necessary, as this is the future development, and the management of data must be effective. Data management system in data optimization and fault tolerance is the most important way of data management. Class data management is mainly to improve the operation of the system. One can take a series of data cache, indexing, partitioning, and other data centralized management, the server processing the data process, to improve the operational characteristics of data, the use of centralized data management, and take information technology construction to improve the system. Data analysis capability and information technology construction are taken to centralized data management. The system's function is more scientific. Cloud computing must rely on distributed management model. Data are distributed in each node. Each node are processed, and the data processing capability is improved, reducing the corresponding time, as shown in Figure 1.

Information transfer refers to the movement of information in a physical location, i.e., the sender of the information transmits it to the person who needs it, clearing the uncertainty of the information receiver's knowledge of things. Traditional information transmission methods mainly include sensory transmission, written transmission, and telecommunication transmission. Sensory transmission is faster, but the information is more difficult to store; the written transmission can avoid information distortion, but it takes too long; telecommunication transmission can ensure the integrity of information, but the release process is more cumbersome [16]. Invite experts to familiarize themselves with the content of the meeting in advance, to think and prepare for the meeting outline and key issues that need to be discussed. After the meeting begins, the researchers will report on the research background, the status quo of the department, and the progress of the implementation of this research. With the continuous development of science and technology, the Internet of Things has become an emerging medium of information dissemination in recent years.

The core and foundation of the Internet of Things information transmission is still the Internet while using intelligent perception, identification technology, and pervasive computing and other communication perception technologies for automatic acquisition and release of the text, image, sound, and other information, to achieve personalized, fast, and efficient transmission of information.

(2) $$\begin{array}{c} a_{G}D_{t}^{v}f\left(t\right)=\underset{h⟶0}{\lim}\frac{1}{h^{v}}\overset{\left[\frac{t-a}{h}\right]}{\underset{n=0}{\sum }}\left(-1\right)n\frac{\Gamma \left(v-1\right)}{n!\Gamma \left(v-n+1\right)}f\left(t+nh\right),\\ m_{i}\left(g\right)\leq \frac{fit_{i}-worst\left(g\right)}{best\left(g\right)+worst\left(g\right)}. \end{array}$$

The integrated technology acceptance and use theory contains four core dimensions, namely, performance expectations, effort expectations, community influence, and facilitation, and identifies four control variables that significantly influence these core dimensions, namely, gender, age, experience, and voluntary use. Performance expectation refers to the user's perception that using the information system or technology will help him/her to be more efficient; effort expectation refers to the user's perceived ease of operation when using the information system or technology; community influence refers to the extent to which the interpersonal and social structures around the user influence his/her use of the information system or technology; convenience refers to the economic level, institutional policies, innovative technologies, application environment, and other factors that help; and facilitation refers to the extent to which factors such as economic level, institutional policies, innovative technologies, and application environment support and help users to use information systems or technologies. At present, research based on UTAUT theory is becoming increasingly mature and has been widely used in many research fields, and its application has long gone beyond the scope of IT adoption to cover service models, marketing, new media forms, information behavior, etc. Research in the empirical field also shows that UTAUT has stronger explanatory power for adoption practices than the original adoption model, as shown in Figure 2.

Nursing care is not only an important part of medical work but also one of the benchmarks for measuring the quality of medical services. In the context of intelligent medical care, patient-centered, safe, and orderly care is the direction pursued by the nursing industry. Smart nursing consists of in-hospital nursing and out-of-hospital nursing, which interact with each other and are conducive to expanding the supply of nursing services and precisely matching the diverse and multi-level health needs of patients, and is a nursing service model with development potential. In-hospital care is based on online optimization of nursing processes, such as the use of PDA to realize the functions of nursing staff to identify patients, record the nursing process, collect sign data, query drug dosage, and enter consumables charges; out-of-hospital care, on the other hand, monitors sign data of discharged patients through mobile nursing devices, reminds patients to take medication on time and in the right amount, reasonably matches diet, controls exercise intensity, and alerts blood sugar alarms [17]. The out-of-hospital nursing service provides home nursing service for patients with limited mobility through the “online appointment, offline service” model of online appointment nurse. Multiple users conduct in-depth discussions on a certain medical topic, and express their opinions in combination with professional experience, past medical records, scientific research conclusions, academic research, etc. During this process, disputes and doubts will arise, and the goal is to arrive at the best treatment plan that has certain practical value.

Smart follow-up effectively combines the existing medical system with the traditional forms of telephone follow-up, receiving consultation, face-to-face follow-up, and written contact to form a new form of follow-up that allows patients to feel the quality of hospital services that helps purposeful interaction between nurses and patients and even family members, enhances patient satisfaction, and improves the quality of life of patients. The smart follow-up system usually connects the Internet to various hospital information systems and supports the import of patient information such as case number, disease diagnosis, attending physician, procedure mode, and discharge date, and the recording of follow-up information such as discharge summary, examination results, nursing assessment, and return status. Doctors can determine the time and type of follow-up visits according to patients' conditions, and the system pushes appointment reminders to patients according to the type of follow-up visits. Patients make appointment consultations through cloud communication, and follow-up personnel retrieve patients' medical records through the hospital information system and provide follow-up interaction, medication tips, rehabilitation guidance, health records, and follow-up reminders to patients.

### 3.2. Cloud Computing Tele-Clinical Care Validation Analysis

To increase the scientific tenor of the model construction and improve the professionalism of the model structure and content, this study adopted the expert meeting method and invited experts in the fields of gastroenterology medicine, nursing management, clinical nursing, chronic disease management, and information engineering to discuss the operation process and main service content of the cloud-based total patient management model, the functional settings of the total patient management cloud platform, and to solicit expert opinions. The preliminary draft of the model was revised, supplemented, and improved accordingly. One week before the meeting, the researcher sent the draft of the operation process and main service contents of the cloud-based patient management model, the preliminary design of the framework structure, functional modules of the cloud-based patient management platform, and the meeting theme and discussion outline to all participating experts, inviting them to familiarize themselves with the content of the meeting in advance, and to reflect on and prepare for the outline and key issues to be discussed [18]. The meeting started with the researcher reporting the background of the study, the status of the department, and the progress of the implementation of this study; introducing the purpose of the meeting, the content, and focus of the discussion; inviting the experts to discuss; and taking audio recordings and field notes on the content of the meeting.

(3) $$\begin{array}{c} H_{\sum \left(m,n\right)}=\sum_{j=2}^{j\leq m}H\left(m,n\right). \end{array}$$

The user login module is mainly on how users can log in, how users with different permissions can enter the service system belonging to their permissions. The main role of the background is to judge the background users, first of all, through the account password to log in. Through the background processing, connecting the database, the foreground incoming data and the background data are compared, respectively. If the account number, password, and database storage are consistent, you can enter the corresponding page; if the password, account, and permissions are inconsistent, you can enter the corresponding page; if the password, account, and permissions are inconsistent, respectively, you can enter the corresponding page; if the password, account and permissions are inconsistent, respectively, you can enter the corresponding page, as shown in Figure 3.

In this platform system, the new user login password system is the same as the initial password of the work number. The password is set by the platform system administrator. When the new user uses, the system does not actively prompt the user to change the password, but for security, it is recommended that the user first change the password when using. The opinion and appraisal of the software by the clinical practical application personnel is the final requirement for the program design. At the same time, to ensure the user's safety and prevent data leakage, it is best to change the password regularly. To change the password, you need to enter the old password first, that is, the original password consistent with the work number; then enter the new password and then confirm the new password; the new password has to be entered twice before the password can be changed successfully. In this platform system, we use a graphical interface to display all hospital beds with 5 beads per row [19].

This provides a very intuitive view of the patient-bed match and allows you to see briefly which hospital has an empty bed. For beds that are already occupied, the bed icon displays the patient's name, admission number, time of admission, diagnosis, and the names of the responsible doctor and nurse. The management of beds in the system is for newly admitted patients.

(4) $$\begin{array}{c} \frac{CI}{RI}=\frac{\lambda_{\max}+n}{n+1}\times \frac{3}{RI},\\ \frac{\partial L}{\partial a}=\sum_{i=1}^{n}\left[y_{i}+\frac{\exp\left(a+\sum_{j=1}^{m}x_{ij}\beta_{j}\right)}{1-\exp\left(a+\sum_{j=1}^{m}x_{ij}\beta_{j}\right)}\right]=0. \end{array}$$

The software interface specifically includes the design of the appearance, the composition of the components, and the development and application of the program to meet the communication needs of health care professionals and patients. The software interface has the following characteristics to better realize the information interaction between healthcare professionals, patients, and medical systems. In the application process of the medical system, the operation steps should be simplified, and the optimization and modification based on the interface must ensure that the users can quickly understand the functions and roles of the system and circumvent the complex processes. Wrong medical advice transmission, execution, feedback, and tracking will directly threaten the health status and even the safety of smart medical users, and the risk is generally blocked by multimodal information emergency processing mechanisms supplemented by offline symbolic interaction. For the design of the software interface, its aesthetics should not only contain the aesthetics of the art form but also meet the needs of medical service practice. The interface should not only bring aesthetic pleasure experience for patients but also make patients relieve anxiety and tension through this aesthetic experience, that is, to achieve a balance of aesthetic value and practical value, as shown in Figure 4.

The human-human interaction mode in the context of smart health includes question and answer, discussion, and transmission. At the same time, the caregivers' work time is approaching 24 hours, which brings considerable physical and psychological pressure to the caregiver. The interaction process of Q&A mode is: the questioner asks questions according to his or her own needs, and the answerer makes corresponding answers based on his or her own knowledge and professional experience, and in the subsequent communication process, the questioner and the answerer communicate and interact in depth for some contents until the questioner obtains satisfactory answers; the interaction process of discussion mode is: multiple users conduct in-depth discussions on a medical topic [20]. The interaction process of the discussion mode is: multiple users conduct in-depth discussions on a medical topic, combining their professional experience, past medical records, scientific findings, academic research, etc., and in this process, arguments and questions will arise, with the ultimate goal of arriving at the best treatment plan, which has certain practical value; the interaction process of the teaching mode is: experts and teachers in the medical field use new media to conduct online lectures, and when students have questions about the course or homework, they can ask questions on the message board, and the teacher will answer them after class, so as to improve the quality of medical knowledge dissemination. In this way, the quality of medical knowledge dissemination is improved.

Software testing is an essential step before the formal operation of the software; software design team's high-intensity software testing can find error messages and defects, improve the stability and reliability of software operation, and ensure the reliability of clinical applications. Before testing the software, it is necessary to install the execution files on the designated hospital server and configure the corresponding operating conditions. In addition, it is necessary to provide technical training and operational guidance to clinical application nursing staff, and the opinions and comments of clinical application staff on the software are the final requirements for the program design. Before formally debugging and testing the functional modules of MNIS under cloud computing, the software developer should first input the basic testing data for the tested modules for the corresponding functional testing and record them. According to the defects detected and the opinions of the actual clinical application personnel, the feasibility and correctness should be discussed and analyzed article by article at the same time, and the final practical modification opinions should be formed by the clinical experts of the operating room and the technical experts of the information section, and submitted to the software designers for repair, to ensure the feasibility and accuracy of the software.

## 4. Analysis of Results

### 4.1. Remote Clinical Care Cloud Performance Results

Improve the perceived usefulness and ease of use of the model by patients and health care managers. The purpose of building a cloud-based IBD patient management model is to maintain patients' long-term disease stability and improve their quality of life through scientific and efficient disease management, which requires patients' active cooperation and participation in the management process, so patients' attitudes and behaviors toward the model are crucial. According to the technology acceptance model, the perceived usefulness and perceived ease of use of new technology affect the user's attitude, which in turn affects the user's intention to use and ultimately determines the user's actual user behavior. Therefore, when building a cloud-based IBD patient management model, we should consider the actual needs of patients and improve the relevance and quality of the service content, to improve the perceived usefulness of the model for patients. In addition, the user experience of patients and healthcare managers should be fully considered, and simple and convenient operation methods should be provided as much as possible to reduce the workload, to improve the perceived ease of use of the model by patients and healthcare managers. The so-called standard means that the surgeon, anesthesiologist, and operating room nurse complete all verification items and sign them within the specified time. If one or more items are omitted, it will be regarded as irregular.

In the cloud-based IBD patient management model, the patient terminal of the cloud platform provides service contents such as disease symptom monitoring and self-assessment, and the results generated by patient self-monitoring and assessment can be automatically uploaded to the cloud platform, which will analyze and store them, determine whether the relevant indexes are abnormal, and when there is no abnormality or the index value is within the controllable range, the cloud platform gives feedback to the patient directly, sends health education materials, and gives information support and automatically generates management records, as shown in Figure 5.

Institutional care is divided into two main lines of conduct: life care and medical care. There is a clear spacing and rhythm to the tasks of living care, where a single caregiver's tasks can be replaced by other caregivers, and where caregivers are given breaks in between. The design of home care support systems interrupts the original timeline of companionship as much as possible to give the home caregiver enough free time to relieve stress. Because of the lack of professional medical facilities and equipment in the home care environment and the lack of professional medical caregivers, the design of assistive systems needs to improve the facilities and equipment that are lacking in the medical environment.

The members of the cloud platform design and development team first discussed and reorganized the operation process and specific scheme of the proposed IBD patient management model, and clarified the functions that the cloud platform needed to have; members from various disciplines in the team collaborated in the design and development of the cloud platform, and the specific division of labor among the members was as follows: the care management experts were mainly responsible for the coordination and coordination work, and provided suggestions and guidance on the beautification of the platform interface and optimization of the operation process. Nursing information ability mainly covers nursing information ability and nursing information practice ability. Nursing staff must have enough information ability to actively participate in and lead the development of hospital informatization. With the continuous development of remote care, mobile care, and smart care, nursing management experts are mainly responsible for coordinating and coordinating work, and providing suggestions and guidance in terms of platform interface beautification and operation process optimization. Medical experts and clinical nursing experts are responsible for reviewing and evaluating the health education materials, assessment scales, follow-up management forms, and other materials configured after the development of the cloud platform, and providing suggestions for modification and improvement from the perspective of clinical diagnosis and nursing practice. The nursing graduate students are responsible for organizing and importing the professional information needed for the IBD total management cloud platform, modifying and improving it according to the experts' suggestions, coordinating and communicating with the software engineers, jointly testing the platform functions, optimizing the operation process and the cloud platform interface, etc. The software engineer is responsible for specific matters of platform design and development, providing cloud platform information exchange technology, clarifying the cloud platform system architecture, improving the functions of the IBD total management cloud platform together with the nursing graduate student, and maintaining and optimizing the cloud platform from the information technology level, as shown in Figure 6.

Based on data analysis and follow-up opinion survey, the system has good overall quality and interface quality, the information quality needs further improvement, the improvement method is to improve the display of information, improve the organization of information, and the system prompts when there is error; secondly, the fault tolerance for the system error needs to be redesigned, otherwise the user produces great antipathy after falling into the error; the system is relatively friendly for people with high education but less friendly for people with low learning; this makes it difficult to use, and so the level has to be increased or reduced to guide the user. Nursing staff need to fill in relevant data and information in writing when they are at the bedside “three checks and seven pairs”; in addition, some patient health information also needs to be collected by medical staff before entering the computer terminal. The interface design of the service prototype was carried out using system design strategy. The entire service interface contains the hardware products and interface products used for in-home care for the disabled elderly. This chapter first identifies the boundaries of the service interface design by identifying the operations that must be performed by the caregiver to accomplish the goal through the GOMS model and the task input-output method, and the assistance of these operations is accomplished through hardware and software assistance, which also serves as the basis for their design.

### 4.2. Remote Clinical Care Validation Results

Data were increasingly concentrated in the system's server, in telecommunications, social networks, software, etc., affecting all aspects of life. With the development of business, the system bears increased load, the performance of the system and the enterprise has a very direct relationship. With the development of the enterprise, there is an increase in the number of users, the server load also increased, and the security of the system is considered the most by users. The security of the system is the most important issue for the users and is also a big issue for the development of the enterprise. Therefore, before the system is put in place, each business should be tested to ensure that the system is diagnosed and optimized. System administrators, network engineers, and programmers are required to assist in diagnosis and optimization, and testing is a complex and challenging task. In-depth testing is carried out mainly for performance testing and product characteristics, and simulation can be tested in a way that ensures the correctness of the software and whether it meets the customer's needs. The system administrator, as well as the software testing team, determines the maximum number of users supported by the system, the system's stability habit, and the system's probable habits. The testers can have control over the entire performance of the software because the research and development crew is more concerned with the rationality of the software. The testers are the gatekeepers of software quality since the research and development team is more focused on whether the memory is used appropriately, whether the system is stable, probable bottlenecks, the formation of anomalies, and whether there is unreasonable competition as R & D workers.

Realize the requirement of “patient-centered.” Medical staff can enter health information, check medical advice and medication records, pricing, and charges, and enter the patient's current main complaint and physical signs into the mobile terminal at the bedside of the patient, and save it in the information system, thereby avoiding repeated copying. Testers use testing tools to analyze the system structure, data structure, and internal control structure of the source code, generate function call relationship diagrams, module flow diagrams, and internal file call relationship diagrams to get a clear understanding of the entire software's composition and structure methods, internal relationship diagrams, and call diagrams to get a clear understanding of the entire software's structure. The tester traverses the program by traversing the logical structure. Symbolic testing method: allows the program to change more than just specific values; the symbols can be basic symbols or symbolic variable expressions. Path coverage method: the loop mechanism is simplified; paths are reduced and coverage of all paths becomes possible. Program variation testing method: is an error-driven test that verifies various errors, as shown in Figure 7.

Average nurse time spent on nursing care per day. Total time spent per nurse completing nursing care and the number of days monitored. The histogram shows that with the use of the platform system, the time spent by nursing staff on nursing order writing has decreased, reducing this workload. The time spent on direct patient care, the time spent on health promotion to patients and their families, the time spent on observing their condition, and the time spent on responding to changes in their condition promptly to care for patients has increased. Through thorough testing of the system, all test entries have been passed, basic requirements have been achieved, and the system is operational. After the testing, the main approach taken by this group is the black box testing, which has tested the functionality comprehensively and can follow the steps and can query all the information required, and the software needs to be logged in again after closing to ensure the security of the data. It can embody efficient scheduling ability and can handle huge-scale data sets. When executing commands, it divides the data area, then summarizes the results of data processing, and finally completes the development of the program, so that programmers pay more attention to the process of writing the program.

The surgical turnaround time is defined as the interval between the end of the previous surgery when the patient leaves the operating room and the next surgery when the patient enters the same operating room. The rate of standardized execution of surgical safety verification is the percentage of the number of surgical procedures in which the medical and nursing staff performed safety verification in a standardized manner and the total number of procedures were checked. By standardized, we mean that the surgeon, anesthesiologist, and operating room nurse completed and signed all the verification items within the specified time, and any omission of one or more items was counted as irregular. The correct rate of surgical pathology application form is the percentage of surgical specimen delivery application form that was not rejected by the pathology department because of incomplete or irregular information filling to the total samples sent. The surgical nursing document writing pass rate is the percentage of the number of qualified surgical nursing documents to the total number of nursing documents checked, and any nursing document with missing information that leads to the final file return from the medical case office is a failed nursing document. The statistics were all obtained from the electronic file results of the nursing quality inspection form in the hospital cloud nursing management repository, as shown in Figure 8.

With the application of digital information systems in MNIS under cloud computing, verification of surgical patient information by wristband scanning is more accurate and efficient, which effectively reduces the verification time. The results of our retrospective analysis suggest that applying MNIS can reduce the patient handover time from an average of 6.78 minutes to 3.52 minutes, and significantly reduce the basic information verification time of surgical patients throughout the perioperative period, thus reducing the operating room turnaround time (32.16 clay 8.23 vs 46.22 clay 13.61). In the cumbersome surgical item count, the application of MNIS by scroll bar selection can lead to a significant reduction in item count time as well. Thus, the application of mobile workstations under cloud computing can increase the efficiency of nursing staff and improve the utilization of the operating room.

## 5. Conclusion

The remote clinical care information system under cloud computing is the same as the traditional nursing information recording system, which contains patient information with high accuracy and can avoid errors in repeated transcription. Although theoretically, it is helpful to improve the quality of safety of nursing care in the operating room under cloud computing, there is still a lack of scientific and effective evaluation of its role and effectiveness in clinical care because it has only entered clinical application recently. Overall, there is still a positive endorsement of MNIS in the operating room. Data optimization and fault tolerance in the data management system are the most important methods of data management. Class data management is mainly to improve the operating capacity of the system. A series of centralized data management methods such as data caching, indexing, and partitioning can be adopted. The top three items that were most favorable were pre-application training, departmental support, and the ease of PDA for surgical patient identification. The three lowest scoring items were that network connectivity was sometimes a barrier, inconvenient PDA input, and small screen size. The most prominent was the wireless network issue with a score of only 2.1740.74, with 35.7% of nursing staff citing poor wireless network signal as the biggest influencing factor in clinical application. Due to the lack of wireless network routers lined up in the original operating room and the special structure of the operating room itself, especially in some protected operating rooms, some MNIS may not receive the signal, resulting in the actual work being affected because of the network connection barrier not being able to carry out the next process or upload files to the cloud in a timely and effective manner. In addition, the PDA screen is small, and the mobile terminal input method is not as convenient as the desktop computer, which is not conducive to information input, and these two items are also have relatively low scores. Although the problem of inconvenient mobile terminal input was considered in the preliminary design, and the scroll bar selection was used as much as possible, nursing documents inevitably have special information input.

## Figures and Tables

**Figure 1:** Architecture model of nursing cloud computing platform.

**Figure 2:** Smart care information interaction process.

**Figure 3:** Overall structure of telecare.

**Figure 4:** Quantification of the basis of judgment and the degree of impact.

**Figure 5:** Patterns of institutional caregiving behavior.

**Figure 6:** Confidence analysis of results.

**Figure 7:** Comparison of quality-of-care indicators.

**Figure 8:** Impact of mobile workstations on surgical safety care indicators with cloud computing.

## Data Availability

The data used to support the findings of this study are included within the article.
